# A Novel Stress State Assessment Method for College Students Based on EEG

**DOI:** 10.1155/2022/4565968

**Published:** 2022-06-07

**Authors:** Li Liu, Yunfeng Ji, Yun Gao, Tao Li, Wei Xu

**Affiliations:** ^1^Jiangsu Vocational College of Information Technology, Wuxi, Jiangsu 214153, China; ^2^Jiangsu Key Laboratory of Media Design and Software Technology (Jiangnan University), Wuxi 214122, China

## Abstract

Stress is an unavoidable problem for today's college students. Stress can arouse strong personal emotional and behavioral responses. Compared with other groups of the same age, college students have a special way of life and living environment. They have complex interpersonal relationships and relatively weak social support systems. At the same time, they also face fierce competition in both academic and employment. However, they lack the skills to deal with the crisis and are reluctant to ask others for help, which leads to a simultaneous increase in mental stress. The pressure on college students mainly comes from study, family, social, employment, society, and economy. When students face multiple pressures from family, school, society, etc., some students are prone to some psychological problems due to their own personality or external environment and other reasons. Therefore, regular assessment of students' stress status is an important means to prevent college students' psychological problems. Considering that in real life, the number of students whose pressure is within the tolerable range is the majority, while the number of students who are under too much pressure is a minority. Therefore, the actual dataset to be identified belongs to a kind of imbalanced data. In this study, an improved extreme learning machine (IELM) is used to improve the performance of the recognition model as much as possible. IELM takes the idea of label weighting as the starting point, introduces the AdaBoost algorithm, and combines its weight distribution with the label weighted extreme learning machine (ELM). During the weight update process, the advantage of the imbalanced nature of multi-label datasets is taken. IELM was used to classify EEG data to determine the stress level of college students. The experimental results demonstrate that the algorithm used in this study has excellent classification performance and can accurately assess students' stress levels. The accurate assessment of stress has provided a solid foundation for the development of students' mental health and has significant practical implications.

## 1. Introduction

College students play an important role in the development and construction of various projects across the country. Their mental health has an impact not only on individual growth and education but also on the country's and society's long-term stability. However, in recent years, college students have experienced psychological crises on occasion, and the subject has grown in prominence, attracting widespread attention from society and university student employees. To address the psychological issues that college students face, we must first comprehend their stress levels. Second, according to the stress condition, the source of psychological stress in college students is precisely evaluated, and the reasons for psychological stress in college students are thoroughly examined. Finally, corresponding intervention strategies are proposed. This is the main connotation of college students' work. Psychological stress is a person's physiological changes and emotional fluctuations caused by changes in the external environment and the stress response of the body. The transition of college students from high school to university is an important turning point from school to society. There are all kinds of stress involved in adapting to a new environment, learning new courses, facing new challenges, and developing new relationships. The sources of psychological pressure on college students mainly include the following aspects: first, the psychological pressure caused by role change and adaptation disorders; second, the learning pressure caused by the change in learning style and weak learning motivation; third, the interpersonal pressure caused by communication difficulties and weak communication skills; fourth, the economic pressure and mental pressure caused by the family's economic difficulties; fifth, the employment pressure caused by the severe employment situation and the fierce competition for talents; sixth, the psychological pressure caused by lack of sexual knowledge and immature concept of love; seventh, the psychological pressure caused by personality and emotional problems; and eighth, psychological pressure caused by personality and emotional problems. The psychological stress of college students directly affects their learning effect and quality of life during their school days. For schools, it is about whether they can produce graduates with excellent mental health and professional quality. In the research on the stress of college students, some scholars believe that college students are a high-stress group. Other studies believe that college students only feel less stress, but the sense of stress and the way of coping with stress are indeed the most important factors that cause college students' mental health problems. If psychological pressure cannot be relieved in time, it may lead to high blood pressure and cardiovascular disease and endanger physical health. Depression, pessimism, and hopelessness accompanying psychological pressure will affect students' academic performance and interpersonal communication. This will lead to college students' life satisfaction and happiness. It can even lead to vicious incidents such as wounding and suicide.

Most of the methods of psychological stress assessment use objective scales. Reference [1] compiled a social readjustment scale (SRRS) containing 43 items, which opened the first instance of using questionnaires to measure stress. Subsequently, some researchers have compiled some stress questionnaires with relatively high reliability and validity, such as the Student Stress Scale prepared in [2] and the Graduate Stress Scale prepared in [3]. Commonly used psychological scales are perceived stress scale (PSS) [4], relative stress scale (RSS) [5], psychological stress measure (PSM) [6], and so on. When the method of filling in the scale is used to evaluate the psychological stress state of the subjects, a large-scale test can be administered in a short period of time, and the test results can be obtained quickly. Compared with other methods, it has the advantages of high efficiency and good scientificity. However, many objective scales used in China are compiled based on the psychological characteristics of Westerners. However, the psychological characteristics of social approval, default tendency, and strong conformity in Chinese people's response to the scale have led to a considerable proportion of students' answers with false elements in the scale test. This affects the authenticity and validity of the questionnaire. Therefore, it is difficult to truly evaluate their psychology and behavior through questionnaires. Due to the shortcomings of the scale test method and the complexity of the respondents' motivation to answer the questions, many scales have already added a certain number of fraud identification questions during the compilation process.

To find a more objective stress assessment method, many scholars began to study stress assessment methods based on physiological signals. Studies have shown that there is indeed a close relationship between psychological stress and brain activity [7]. In particular, when negative emotions appear, the activity of the right hemisphere of the brain is abnormally active [8]. Therefore, scholars have begun to boldly hypothesize that the relative activity of EEG on the right side of the brain predicts changes in psychological stress and a higher risk of mental illness [9]. Based on this conclusion, many EEG-based stress recognition studies have appeared one after another. Reference [10] studied a number of subjects who faced examination pressure and found that the subjects' right forehead EEG activity was more intense under high-intensity examination pressure. Reference [11] studied the stability of prefrontal EEG asymmetry for detecting psychological stress and depression levels, and the results showed that resting EEG *α* wave asymmetry could be used as a reliable indicator for detecting stress and depression levels. However, some literature studies also pointed out that gender and age differences have a greater impact on the study of psychological stress [12]. Reference [13] proposed that gender differences in prefrontal asymmetry and negative emotion processing may be related to human genes.

To sum up, we found that the existing researches on stress state recognition are based on different types of data such as scales, EEG signals, ECG signals, speech signals, video signals, and facial expressions. The evaluation models used are also different for different data types. Common models are mainly based on machine learning [14–16] and deep learning [17–19]. Because the physiology is more realistic, this study mainly chooses the data based on the physiological signal to identify the stress state. Among the physiological data, EEG and ECG are the most common. Considering that the ECG signal acquisition equipment requires multiple electrodes to collect signals, even a single-lead wearable product is not very convenient. In contrast, EEG signals are easier to acquire, and the signals are sensitive, which can quickly reflect changes in pressure. Therefore, this study chooses EEG as the data type used in the research. In the selection of the recognition model, considering that although the recognition rate of the deep learning algorithm is better, its model training time and high requirements for the hardware performance of the device are high, and the model has a lot of parameters. In this study, the theory is simple and easier to implement the machine learning algorithm. Considering that in real life, the number of students whose pressure is within the tolerable range is the majority, while the number of students who are under too much pressure is a minority. Therefore, the actual dataset to be identified belongs to a kind of imbalanced data. In this study, IELM is used to improve the performance of the recognition model as much as possible. IELM takes the idea of label weighting as the starting point, introduces the AdaBoost algorithm, and combines its weight distribution with the label weighted extreme learning machine. During the weight update process, the advantage of the imbalanced nature of multi-label datasets is taken. IELM was used to classify EEG data in order to determine the stress level of college students. The experimental results demonstrate that the algorithm used in this study has excellent classification performance and can accurately assess students' stress levels.

## 2. EEG-Based Stress Detection

### 2.1. The Relationship between EEG and Students' Stress State

Stress, pleasure, focus, etc., are all related to human emotional thinking. The brain controls human thoughts and emotions. When the brain deals with emotion-related issues, the amygdala, orbitofrontal cortex, anterior cingulate cortex, insula, nucleus accumbens, thalamus, and ventral tegmental area of the brain all respond differently to specific emotions. For example, the anterior cingulate cortex responds when we make a decision about something in a happy or sad emotional state. The nucleus accumbens becomes active when we anticipate a reward or something good will happen. When something disgusts us, the insula becomes very active. When these areas are stimulated and activated, neurons in the cerebral cortex are stimulated to generate action potentials. When the cells are stimulated by the impulse, the pyramidal cells will be depolarized, forming a potential difference and generating an electric current. After the electrodes are placed on the scalp, and after amplification, the EEG signal can be collected and an EEG can be drawn. People divide EEG signals into *δ*, *θ*, *α*, *β*, and *γ* frequency bands according to different frequency bands. The descriptions of brain waves in each frequency band are shown in Table 1.

Research has shown that when we blink or think, *α* waves instantly disappear and reappear, and *β* waves become very active and have high amplitudes. *γ* is very sensitive to emotional changes and cognitive learning. When we are tired and sleepy, *θ* waves begin to appear and become active. To sum up, it can be found that the generation and activity of different brain waves can intuitively reflect the current activity state of students. Therefore, by studying the brain wave signals of these frequency bands, we can analyze the emotional state of college students in the process of study and life and then analyze the stress state of students.

### 2.2. EEG-Based Stress Assessment

Figure 1 shows the stress assessment process based on EEG signals.

As shown in Figure 1, the first step is to collect EEG data. EEG data collected are all from the freshman to third-year students of our school. Since EEG is a very weak physiological electrical signal, its amplitude can generally only reach the order of microvolts. Therefore, during the acquisition process, various noises generated by different reasons such as the surrounding environment, eye movement signals, and EMG signals are easily mixed into the collected EEG, resulting in poor experimental results. Therefore, to ensure EEG's purity, it is often necessary to perform preprocessing such as denoising the EEG before analyzing the EEG data.

To reduce the data dimension and facilitate subsequent classification processing, feature extraction operations on the preprocessed data are usually required. At present, the research on EEG signal features mainly focuses on linear features, such as extracting the frequency, power, and other features of EEG signals by means of the Fourier transform. However, the structure of the human brain is more complex, and nonlinear features often have better performance. Generally, the linear and nonlinear characteristics are shown in Table 2.

A stress state recognition model is trained based on the EEG training dataset. The algorithm used is the IELM algorithm given in Section 3. The performance of the trained model is validated using the test dataset. The higher the classification accuracy of the sample, the better the model.

## 3. Imbalanced Extreme Learning Classification Algorithm

### 3.1. Weighted Extreme Learning Algorithm

For class-balanced tasks, weighted extreme learning is particularly successful. However, it has two drawbacks. First, as the size of the training set grows, so does the time complexity. The second issue is a lack of mistake compensation flexibility. Reference [20] developed a marker-weighted extreme learning machine based on the concept of cost-sensitive learning to address the drawbacks of this technique. By increasing the expected output value of minority class labels, label-weighted extreme learning machines improve the training error tolerance of minority class cases. Furthermore, because it does not use a weight matrix in the optimization method, it has the same time complexity as standard ELM.

(1) $$\begin{array}{c} L_{ELM}=\frac{1}{2}{\left\|\beta \right\|}^{2}+\gamma \frac{1}{2}W\overset{N}{\underset{i=1}{\sum }}{\left\|\tau_{i}\right\|}^{2},\\ h\left(x_{i}\right)\beta =t_{i}^{T}-\tau_{i}^{T},\\ i=1,2,\ldots ,n. \end{array}$$

Assume that the expected matrix *T* has *m* rows and *n* columns, where *m* is the number of categories and *n* is the number of training set samples. The penalty factor is *γ*. The output layer weight to be solved is denoted by *β*. *W* is an *n*-dimensional diagonal matrix. Each diagonal element's value corresponds to the penalty factor regulation parameter of the corresponding sample.

*τ*_*i*_=[*τ*_*i*1_, *τ*_*i*2_,…, *τ*_*im*_] represents the training error vector corresponding to the sample *x*_*i*_ on all output nodes. The expression for *T* is as follows:

(2) $$\begin{array}{c} T=\left[\begin{array}{cccc} \begin{array}{c} t_{11}\\ t_{21}\\ \vdots \\ t_{m1} \end{array} & \begin{array}{c} t_{12}\\ t_{22}\\ \vdots \\ t_{m2} \end{array} & \begin{array}{c} \cdots \\ \cdots \\ \ddots \\ \cdots \end{array} & \begin{array}{c} t_{1N}\\ t_{2N}\\ \vdots \\ t_{mN} \end{array} \end{array}\right]. \end{array}$$

For the setting of label weights in two-class and multi-class classification problems, [20] provides two weight distribution methods, as follows:

(3) $$\begin{array}{c} t_{ij}=\left\{\begin{array}{cc} \Delta \text{major}\left(\text{num}\right)/\Delta \left({\text{num}}_{i}\right), & \text{if }x_{j}\in {\text{num}}_{i},\\ -1, & \text{if }x_{j}\notin {\text{num}}_{i}, \end{array}\right.\\ t_{ij}=\left\{\begin{array}{cc} \sqrt[{2}]{\Delta \text{major}\left(\text{num}\right)/\Delta \left({\text{num}}_{i}\right)}, & \text{if }x_{j}\in {\text{num}}_{i},\\ -1, & \text{if }x_{j}\notin {\text{num}}_{i}. \end{array}\right. \end{array}$$

where Δ(num_*i*_) is the number of samples from the *i*th class in the training set and Δmajor(num) is the number of samples from the majority class. Two weight distribution methods are provided:

(4) $$\begin{array}{c} t_{ij}=\left\{\begin{array}{cc} ∼\Delta major\left(num\right)/\Delta \left(num_{i}\right), & if\;x_{j}\in num_{i},\\ -1, & if\;x_{j}\notin num_{i}, \end{array}\right.\\ t_{ij}=\left\{\begin{array}{cc} \sqrt[{2}]{∼\Delta major\left(num\right)/\Delta \left(num_{i}\right)}, & if\;x_{j}\in num_{i},\\ -1, & if\;x_{j}\notin num_{i}, \end{array}\right.. \end{array}$$

The weights of the majority class samples remain unchanged in the above weight distribution method, while the weights of the minority class samples are increased. The greater the class imbalance ratio, the greater the weight ratio between the minority and majority classes. The following steps are taken by the weighted extreme learning (Algorithm 1).

### 3.2. AdaBoost Algorithm

In ensemble learning, according to the different ways of generating base learners, it can be divided into serial ensemble learning algorithms represented by boosting [21] and parallel ensemble learning algorithms represented by bagging [22]. Among the boosting learning paradigms, the AdaBoost algorithm is the most famous, originally proposed by Freund and Schapirel in 1997.

Suppose **X** is a set containing *n* training samples for training an AdaBoost classifier. In the AdaBoost algorithm, the importance of each base classifier *H*_*i*_ depends on its error rate *ε*_*i*_:

(5) $$\begin{array}{c} \varepsilon_{i}=\frac{1}{n}\left[\sum_{j=1}^{n}w_{j}F\left(H_{i}\left(x_{j}\right)\neq y_{j}\right)\right], \end{array}$$

where *F* is the indicator function. If the condition is true, it takes the value 1; otherwise, it is 0. Through the above formula, the importance weight of the base classifier *H*_*i*_ is given as follows:

(6) $$\begin{array}{c} \varsigma_{i}=\frac{1}{2}\ln\left(\frac{1-\varepsilon_{i}}{\varepsilon_{i}}\right). \end{array}$$

It can be seen that when the error rate *ς*_*i*_ is close to 0, *w*_*i*_^(*j*)^ corresponds to a large positive value. When the error rate is close to 1, *w*_*i*_^(*j*)^ corresponds to a large negative value.

(7) $$\begin{array}{c} w_{i}^{\left(j+1\right)}=\frac{w_{i}^{\left(j\right)}}{S_{j}}\times e^{-\varsigma_{j}L_{j}\left(x_{i}\right)y_{i}}\\ =\frac{w_{i}^{\left(j\right)}}{S_{j}}\times \left\{\begin{array}{c} e^{-\varsigma_{j}}\text{ if }H_{j}\left(x_{i}\right)=y_{i},\\ e^{\varsigma_{j}}\text{ if }H_{j}\left(x_{i}\right)\neq y_{i}, \end{array}\right. \end{array}$$

where *S*_*j*_ is a normalization factor to ensure that ∑_*i*_*w*_*i*_^(*j*)^=1.

Through the above weight update formula, it is possible to increase the weight of the misclassified samples in the previous round and reduce the weight of those that have been correctly classified. The AdaBoost algorithm's execution steps are as follows (Algorithm 2).

### 3.3. IELM

Reference [23] weights the tokens to increase the expected output of minority class samples. By improving the training error tolerance of the minority class samples, the overall training error of the minority class is similar to that of the majority class in the global training error. In this way, the class imbalance problem is solved. Since the label weight only changes the expected output size and does not change the original optimization formula of the extreme learning machine, the time complexity does not change. However, this algorithm also has certain shortcomings. For example, the algorithm uses human experience to set the weights, which lacks flexibility. The core idea of the AdaBoost algorithm is to change the distribution of samples by modifying the weight of the samples, so that the classifier gradually focuses on those samples that are easy to be misclassified. In this way, the quality of the classification model is maximized. In the label weighting process, larger weights are often assigned to those important samples to avoid misclassification. The above two strategies have the same idea. Based on the inspiration of this idea, this study combines AdaBoost with a labeled weighted extreme learning machine. To efficiently deal with multi-label imbalanced data, the algorithm used improves the two key aspects of AdaBoost's initial weight setting and weight distribution update. The improved model always considers the inherent imbalance characteristics of multi-label and adjusts the size of the weights directionally.

#### 3.3.1. Adjust the Initial Weight

For single-label classification problems, the weight distribution reflects the relative importance of the samples. Training samples that are often misclassified tend to receive larger weights than correctly classified samples. For multi-label classification problems, the weight distribution can reflect the relative importance of the labels. Therefore, the object of weight setting is the marker. The traditional weight setting method is to use the method of evenly distributing the weight. If the data distribution is unbalanced, the weight can be increased by updating the weight in the iterative process and adjusting the minority class adaptively. In fact, the unbalanced degree of the data can be considered. Giving the minority class a higher weight and the majority class a lower weight will inevitably cause the model to converge faster.

Assuming that the multi-label data *S*={(*x*_*i*_, *Y*_*i*_)*|i*=1,2,…, *n*} are a training set containing *n* samples, *V*={*v*_*j*_*|*1,2,…, *c*} represents a label set with *c* categories, where *xi* is the feature vector of the *i*th sample, and *Y*_*i*_⊆*V* is its associated label set.

Reference [24] proposed an intra-marker imbalance measure, which has been widely used. For the *j*th marker, *S*_*j*_^+^={(*x*_*i*_, +1)*|y*_*j*_ ∈ *Y*_*i*_,  1 ≤ *i* ≤ *n*} represents the positive class sample, *S*_*j*_^−^={(*x*_*i*_, −1)*|y*_*j*_ ∉ *Y*_*i*_,  1 ≤ *i* ≤ *n*} represents the negative class sample, and the imbalance rate of the *j*th marker is as follows:

(8) $$\begin{array}{c} R_{j}=\frac{\max\left(\left|S_{j}^{+}\right|,\left|S_{j}^{-}\right|\right)}{\min\left(\left|S_{j}^{+}\right|,\left|S_{j}^{-}\right|\right)}. \end{array}$$

The initial weight is set as an asymmetric matrix *W* according to the imbalance ratio, and **W** contains *n* rows and *c* columns, representing *n* samples and *c* markers, respectively. The *j*th token value of the *i*th sample is as follows:

(9) $$\begin{array}{c} t_{ij}=\left\{\begin{array}{cc} \sqrt{\left(R_{j}\right)}, & \text{if }x_{i}\in {\text{num}}_{j},\\ 1, & \text{if }x_{i}\in {\text{num}}_{j}, \end{array}\right.. \end{array}$$

(10) $$\begin{array}{c} W_{ij}=\frac{t_{ij}}{p_{i}}, \end{array}$$

where *p*_*i*_ is the normalization factor, and its function is to constrain the sum of the weights of the markers to be 1. The square root of *R* is chosen here because the imbalance ratio in the multi-label is relatively high, and direct use will cause the weight of positive samples to be much larger than the weight of negative samples, making the model fall into the other extreme.

#### 3.3.2. Weight Update

In this study, the purpose of setting asymmetric weight distribution is to make AdaBoost always focus on the imbalance problem within the label. In the iterative process, if the weights are updated in the usual way, the model cannot keep focusing on the multi-label imbalance problem. Therefore, this study updates the weights separately for each category of each token. For the lth label, its *j*th class error rate is calculated as follows:

(11) $$\begin{array}{c} \varepsilon =\sum_{x_{i}\in \text{class }j:H{\left(x_{i}\right)}^{l}\neq Y_{i}^{l}}S_{t}\left(x_{i}\right), \end{array}$$

where *H* represents the base classifier used by the model and *H*(*x*_*i*_)^*l*^ represents the output of the base classifier on the *l*th token of the sample instance **x**_*i*_.

(12) $$\begin{array}{c} \varsigma^{lj}=\frac{1}{2}\ln\left(\frac{\sum_{x_{i}\in \text{ class }j:H{\left(x_{i}\right)}^{l}=Y_{i}^{l}}S_{t}\left(x_{i}\right)}{\sum_{x_{i}\in \text{ class }j:H{\left(x_{i}\right)}^{l}\neq Y_{i}^{l}}S_{t}\left(x_{i}\right)}\right). \end{array}$$

When the error rate is close to 0, *ς* corresponds to a large positive value. When the error rate is close to 1, *ς* corresponds to a large negative value. The calculation formula of the weight *W* of the *t* + 1th round is as follows:

(13) $$\begin{array}{c} W_{\text{t}+1}^{lj}\left(x_{i}\right)=\frac{W_{t}\left(x_{i}\right)\exp\left(-\varsigma_{t}^{lj}F\left(H\left(x_{i}\right),j\right)\right)}{p_{t}^{lj}}, \end{array}$$

where *F*(·) is an indicator function, and the role of p_*t*_^*lj*^ is to ensure ∑*w*_*t*+1_^*lj*^(*x*_*i*_)=1/2*q* at this time. The weight calculation formula of the entire trainer is as follows:

(14) $$\begin{array}{c} \varsigma =\frac{1}{2}\ln\left(\frac{\sum_{l}\sum_{i:H{\left(x_{i}\right)}^{l}=Y_{i}^{l}}S_{t}\left(x_{i}\right)}{\sum_{l}\sum_{i:H{\left(x_{i}\right)}^{l}\neq Y_{i}^{l}}S_{t}\left(x_{i}\right)}\right). \end{array}$$

#### 3.3.3. IELM Algorithm Execution Steps

The IELM algorithm's execution steps (Algorithm 3) are as follows.

## 4. Experiment

### 4.1. Experimental Data Collection

To ensure that the experiment is not affected by factors such as the subject's physical health, other disturbances are minimized as much as possible. Therefore, before this experiment, we learned about the physical condition and basic information of each subject by means of a questionnaire, including the subject's name, age, gender, physical condition, academic status, family status, and the relationship with classmates and teachers. In the questionnaire, subjects are required to check the stress self-evaluation items. The table design of the questionnaire is shown in Table 3.

To better collect EEG without external interference, subjects were first allowed to fall asleep in a quiet environment. When the subject entered deep sleep, the subject's EEG was collected. A total of 35 questionnaire data and EEG data were collected from freshmen to junior college students. These data are simply screened according to the questionnaires filled in by the subjects. For example, when there is a large deviation between the subjects' emotions and the expected emotions of the videos watched, or the subjects are not in the state at all when watching the videos, this set of data will be discarded. Finally, 90 valid samples and 360 EEG fragments were screened out.

### 4.2. Multifeature Combination Experiment

There are many features of EEG data. This study mainly extracts four features: Hurst index (P1), volatility index, sample entropy, and permutation entropy. The collected EEGs were classified using radial basis neural network (RBFNN) and IELM. The number of categories is 3, which are high stress, average stress, and low stress. The two algorithms run 10 times on each rhythm to get the average classification accuracy.  Table 4 and Figure 2 show the experimental results based on the ELM algorithm.  Table 5 and Figure 3 show the experimental results based on the IELM algorithm.

Figures 2 and 3 show that, regardless of classifier, the fluctuation index has the best classification effect, followed by the Hurst index and permutation entropy, and the worst is sample entropy. This demonstrates that different types of features contribute to the classification results at different rates.  Figure 4 depicts the classification accuracy of various classifiers from four different perspectives.

As can be seen from Figure 4, under a single feature, the classification accuracy of the IELM algorithm under a single feature is higher than that of the ELM. To resolve the optimal combination of multiple features to improve the classification recognition rate of EEG, in this study, a linear weighting formula is given to obtain the weight of each EEG feature. The weight calculation formula is as follows:

(15) $$\begin{array}{c} w_{i}=\frac{f_{i}}{f_{1}+f_{2}+f_{3}+f_{4}},\\ \text{s.t}.1\leq i\leq 4,\;0\leq w_{i}\leq 1, \end{array}$$

where *f*_*i*_ is the classification recognition rate based on the *i*th EEG feature and *w*_*i*_ is the weight of the feature *f*_*i*_. The data in Table 5 are substituted into equation (15), and the calculated feature weights are shown in Table 6.

The weights of the combined features under each frequency band can be obtained from the data in Table 6, and the feature combination formulas under 5 frequency bands are as follows:

(16) $$\begin{array}{c} F_{\alpha }=0.2556P1+0.2673P2+0.2363P3+0.2408P4, \end{array}$$

(17) $$\begin{array}{c} F_{\beta }=0.2582P1+0.3007P2+0.2212P3+0.2198P4, \end{array}$$

(18) $$\begin{array}{c} F_{\gamma }=0.2927P1+0.2913P2+0.1965P3+0.2195P4, \end{array}$$

(19) $$\begin{array}{c} F_{\delta }=0.2281P1+0.2808P2+0.2250P3+0.2661P4, \end{array}$$

(20) $$\begin{array}{c} F_{\theta }=0.2653P1+0.3084P2+0.2033P3+0.2230P4. \end{array}$$

It can be seen from the experimental data in Table 6 that the weights of the Hurst index and fluctuation index are higher than the remaining two features in the five rhythm species. This shows that these two features show more superior performance in the task of stress assessment. The EEG data of the two feature combinations were classified separately using IELM.  Table 7 and Figure 5 give the classification results.

It is clear from the experimental results shown in Table 7 and Figure 5 that for the same classification model, the accuracy of the weighted feature combination is significantly higher than that of the unweighted feature combination. This shows that the introduction of feature weighting strategy can improve the classification performance of EEG. The reason is that different types of features have different degrees of activity for classification. Based on the weighting formula given in this study, the features with high activity are given a large weight, and the features with low activity are given a small weight, so that the result is optimal.

### 4.3. Classification Model Experiment

Following the selection of the feature combination method, multiple comparison models are introduced to validate the performance of the classification model used in this study. They are support vector machine (SVM), linear support vector machine (linear SVM), radial basis neural network (RBFNN), random forest (RF), and ELM. Since a single indicator of recognition accuracy cannot fully characterize the performance of the recognition model, this study also introduces the recall indicator to evaluate the model. The experimental results obtained by different classification models are shown in Table 8 and Figure 6.

By observing the experimental results shown in Table 8 and Figure 6, the following experimental conclusions can be obtained:

1. Among various classification models, the experimental results obtained by the ELM model are relatively better, close to 0.8. This is one of the reasons why this study chooses ELM as the basic algorithm. When the label weighting and AdaBoost are introduced to optimize the traditional ELM, the experimental results obtained by IELM have been greatly improved. Compared with ELM, its accuracy is improved by 10.25%. This proves the effectiveness of the improved strategy in this study.
2. A single indicator is not enough to illustrate the superiority of the model used, so the recall indicator is introduced in the experiment. Compared with SVM, linear SVM, RBFNN, RF, and ELM, the recall rate of the IELM algorithm used is increased by 36.8%, 32.99%, 25.25%, 36.14%, and 15.95%, respectively. The model in this study has been greatly improved in terms of recall rate. This demonstrates the robustness of the algorithm used in this study.

## 5. Conclusion

Psychological stress has a great impact on human health. The role of early detection and intervention of psychological stress in preventing mental diseases cannot be ignored. However, in terms of stress identification methods, traditional psychological tools such as self-rating scales are highly subjective, and hormone measurement cannot be widely promoted due to its invasiveness and other limitations. The current noninvasive objective evaluation method is still in the research stage. In this study, EEG was selected to assess the psychological stress state of college students. The experiment finally determined the EEG data of 90 students to be used in the experiment. There are 30 students in each grade of freshman, sophomore, and junior. According to the stress assessment obtained from the questionnaire, 7% of the freshmen were under great stress, 43% were under average stress, and 50% were under little stress. In the sophomore year, 13% were under great stress, 47% were under average stress, and 40% were under less stress. In the third grade, 20% were under great stress, 53% were under average stress, and 27% were under less stress. In general, 14% were under high stress, 47% were under moderate stress, and 39% were under less stress. Among the results obtained by the stress state assessment method based on EEG identification, 12% were under high stress, 46% were under moderate stress, and 42% were under low stress. The stress assessment results obtained using the model used in this study are relatively close to the questionnaire results. This demonstrates that the method described in this study has a certain reference value. However, this study has some limitations. First, whether the self-made questionnaire can collect the most real stress state data needs further research. Second, the number of pressure states used in the experiment is 3, and the division range is relatively general. Future plans are to explore more objective and rigorous data collection methods and optimize the number of stress classifications.

## Figures and Tables

**Figure 1:** EEG-based stress assessment process.

**Figure 2:** Comparison chart of classification accuracy based on ELM under four features.

**Figure 3:** Comparison chart of classification accuracy based on IELM under four features.

**Figure 4:** Classification accuracy of 4 features. (a) Hurst index. (b) Fluctuation index. (c) Sample entropy. (d) Permutation entropy.

**Figure 5:** Comparison chart of classification accuracy under different feature combinations.

**Figure 6:** Accuracy and recall of different classification models.

**Algorithm 1:** LW-ELM algorithm.

**Algorithm 2:** AdaBoost algorithm.

**Algorithm 3:** IELM algorithm.

**Table 1:** Brain wave band details.

Name	Frequency (Hz)	Location	Generated time
*δ*	0.5 < 4	Forehead in adults, back of brain in children	Occurs mostly in the brains of infants, but also occurs when adults are in deep sleep, coma, or anesthesia
*θ*	4–7	Brain regions unrelated to hand function	Occurs in young children and adolescents, but also in adults who are tired but conscious
*α*	8–15	The back of the brain, the resting state is concentrated in the center	Relaxed/contemplative state with eyes closed
*β*	16–31	The brain is symmetrically distributed on both sides, with a prominent forehead	Positive thinking, focus, vigilance, anxiety
*γ*	32–45	Somatosensory cortex	Short-term memory, hearing, and touch, multisensory processing

**Table 2:** Linear and nonlinear characteristics of EEG.

Feature type	Feature name
Linear feature	Full-band center frequency, Hjorth parameter, peak-to-peak, variance, slope, kurtosis
Nonlinear feature	CO complexity, correlation dimension, power spectral entropy, full-band power spectral entropy, Shannon entropy, Kolmogorov entropy

**Table 3:** Stress self-assessment form.

Subject number				
Gender	Male ☐		Female ☐	
Grade	1 ☐	2 ☐		3 ☐
Study stress	1 ☐	2 ☐		3 ☐
Life pressure	1 ☐	2 ☐		3 ☐
Family stress	1 ☐	2 ☐		3 ☐
Overall pressure	1 ☐	2 ☐		3 ☐

**Table 4:** Classification accuracy based on ELM under four features.

Feature	*α*	*β*	*γ*	*δ*	*θ*
Hurst index	0.7122	0.6945	0.7342	0.5898	0.6342
Fluctuation index	0.8098	0.8120	0.7788	0.7556	0.7861
Sample entropy	0.6541	0.5987	0.5062	0.6012	0.5142
Permutation entropy	0.7193	0.6298	0.5865	0.7181	0.5880

**Table 5:** Classification accuracy based on IELM under four features.

Feature	*α*	*β*	*γ*	*δ*	*θ*
Hurst index	0.7778	0.7624	0.7997	0.6175	0.7037
Fluctuation index	0.8134	0.8878	0.7959	0.7602	0.8178
Sample entropy	0.7190	0.6530	0.5368	0.6091	0.5392
Permutation entropy	0.7327	0.6490	0.5997	0.7204	0.5914

**Table 6:** Details of each feature weight.

Feature	*α*	*β*	*γ*	*δ*	*θ*
Hurst index	0.2556	0.2582	0.2927	0.2281	0.2653
Fluctuation index	0.2673	0.3007	0.2913	0.2808	0.3084
Sample entropy	0.2363	0.2213	0.1965	0.2250	0.2033
Permutation entropy	0.2408	0.2198	0.2195	0.2661	0.2230

**Table 7:** Classification accuracy under different feature combinations.

Feature combination	*α*	*β*	*γ*	*δ*	*θ*
Without weighted feature combination	0.8210	0.8932	0.8090	0.7881	0.8012
With weighted feature combination	0.8340	0.9001	0.8559	0.8293	0.8749

**Table 8:** Experimental results of different classification models.

Index/model	SVM	Linear SVM	RBFNN	RF	ELM	IELM
Accuracy	0.6275	0.6598	0.7609	0.7567	0.7912	0.8728
Recall	0.6515	0.6702	0.7122	0.6547	0.7687	0.8913

## Data Availability

The labeled dataset used to support the findings of this study is available from the corresponding author upon request.
